The article "Lightweight Multireceptive Field CNN for 12-Lead ECG Signal Classification" was published in 2022. Journal: Comput Intell Neurosci.

# Lightweight Multireceptive Field CNN for 12-Lead ECG Signal Classification

**DOI:** 10.1155/2022/8413294

**Published:** 2022-08-08

**Authors:** Degaga Wolde Feyisa, Taye Girma Debelee, Yehualashet Megersa Ayano, Samuel Rahimeto Kebede, Tariku Fekadu Assore

**Affiliations:** ^1^Ethiopian Artificial Intelligence Institute, P.O. Box 40782, Addis Ababa, Ethiopia; ^2^Department of Computer Engineering, Addis Ababa Science and Technology University, P.O. Box 120611, Addis Ababa, Ethiopia; ^3^Department of Electrical and Computer Engineering, Debre Berhan University, Debre Berhan 445, Ethiopia; ^4^Yekatit 12 Hospital Medical College, Addis Ababa, Ethiopia

## Abstract

The electrical activity produced during the heartbeat is measured and recorded by an ECG. Cardiologists can interpret the ECG machine's signals and determine the heart's health condition and related causes of ECG signal abnormalities. However, cardiologist shortage is a challenge in both developing and developed countries. Moreover, the experience of a cardiologist matters in the accurate interpretation of the ECG signal, as the interpretation of ECG is quite tricky even for experienced doctors. Therefore, developing computer-aided ECG interpretation is required for its wide-reaching effect. 12-lead ECG generates a 1D signal with 12 channels among the well-known time-series data. Classical machine learning can develop automatic detection, but deep learning is more effective in the classification task. 1D-CNN is being widely used for CVDS detection from ECG datasets. However, adopting a deep learning model designed for computer vision can be problematic because of its massive parameters and the need for many samples to train. In many detection tasks ranging from semantic segmentation of medical images to time-series data classification, multireceptive field CNN has improved performance. Notably, the nature of the ECG dataset made performance improvement possible by using a multireceptive field CNN (MRF-CNN). Using MRF-CNN, it is possible to design a model that considers semantic context information within ECG signals with different sizes. As a result, this study has designed a multireceptive field CNN architecture for ECG classification. The proposed multireceptive field CNN architecture can improve the performance of ECG signal classification. We have achieved a 0.72 *F*_1_ score and 0.93 AUC for 5 superclasses, a 0.46 *F*_1_ score and 0.92 AUC for 20 subclasses, and a 0.31 *F*_1_ score and 0.92 AUC for all the diagnostic classes of the PTB-XL dataset.

## 1. Introduction

ECG is a medical device used to monitor the heart's electrical activity and rhythm of the heart [1]. The electrical pulses produced by the heart organ each time the heart beats are detected by the sensors attached to the skin, and the device gives a voltage versus time electrical activity of the heart [2]. In 12-lead ECG, there are 12 directions from which an electrical signal or impulse generated by the heart can be measured [3]. The ECG signal generated by each lead contains waves, intervals, segments, and one complex [4], as shown in Figure 1. The waves indicate a specific electrical event, a negative or positive deflection from the baseline. ECG waves include the P wave, Q wave, R wave, S wave, T wave, and U wave. The period between two specific ECG events is referred to as the interval. The PR interval, QRS interval (also known as QRS duration), QT interval, and RR interval are routinely observed on an ECG. The segment is the distance between two specific locations on an ECG that should be at the same amplitude as the baseline (not negative or positive). The PR, ST, and TP segments are the three segments of an ECG. The QRS complex is the only one on an ECG, consisting of many grouped waves. On the other hand, the QRS complex includes Q, R, and S waves and represents ventricular depolarization. The T wave indicates ventricular repolarization after the QRS complex.

During interpretation, doctors examine the ECG signals printed on the ECG paper and look for the anomalies that could appear in the signal wave, interval segment, and complex. Cardiovascular diseases are related to those changes that happen in the signal. However, cardiologist shortage is a challenge in both developing and developed countries. Moreover, the experience of a cardiologist matters in the accurate interpretation of the ECG signal, as the interpretation of ECG is quite tricky even for experienced doctors. Therefore, developing computer-aided ECG interpretation is required for its wide-reaching effect. Early computer analysis tools used deterministic algorithms to interpret ECG data using logical decision rules devised by expert ECG readers. The algorithms employed narrowly defined cutoff points to see if they met a decision criterion. However, this approach was not practical across individuals with varying QT intervals [5]. Since the 1980s, computerized ECG data classification has incorporated probability theory and statistics. These include Bayesian analysis, multivariate statistics, and, more recently, ML approaches such as SVMs, neural networks, and deep learning methods.

The remarkable advancement of medical image classification using conventional machine learning and deep learning algorithms indicates the feasibility of borrowing the same concept for computer-aided time-series signal classification. In the classical machine learning approach, time-domain feature extraction is performed, and the result is fed to classifiers like KNN, SVMs, neural networks, and so forth [6–9]. On the other hand, in deep learning, a raw time-series signal is given as input to the deep learning model. We generally talk about 2D-CNN for image classification when we refer to CNN. However, there are two other types of CNN, which are 1D-CNN and 3D-CNN. The exact process used for 2D-CNN image analysis can be harnessed for 1D data sequences, such as acceleration and gyroscopic data for human activity recognition, bearing fault analysis from vibration signals, and audio classification [10–12]. The model extracts features from observations by convolving the signal with 1D filters along one dimension and generating feature maps.

The advantage of using 1D-CNNs for sequence classification is that they can learn from raw time-series data straightforwardly and do not require domain expertise to engineer input features manually [13–15]. The model can acquire knowledge about the internal representation of the time-series data. Theoretically, it achieves comparable performance to model fit on a manually engineered dataset feature. The input and output of 1D-CNN are two-dimensional (width of the data and its channel). For example, the 12-lead ECG signal has 12 channels with N signal length/width. On sequence processing problems, 1D-CNNs can be competitive with RNNs, usually, at a lower computational cost [16]. 1D-CNNs have recently been successfully employed for audio generation and machine translation, primarily with dilated kernels [17, 18]. Aside from these specific accomplishments, small 1D-CNNs have long been known to be a fast alternative to RNNs for simple tasks like text classification and time-series forecasting [19]. What makes CNN work well for time-series signals is the windowed convolution that produces a receptive field. The receptive field is a portion of a sensory space that can give rise to a neuronal response when stimulated, or it is a portion of an input signal that can enable a single neuron [20]. It can also be defined as a region in an input that produces a feature map when convolved with a filter. Kernels in CNN access this region and make the feature map. The receptive field has a direct relationship with the size of the filter. The larger the kernel size is, the larger the receptive field will be. Thus, a small receptive field may not recognize extensive features in the signal. On the contrary, an unnecessarily sizeable receptive field would result in more parameters that are not useful in the feature extraction. That is why multiscale approaches are usually seen in object detection.

The main task of artificial intelligence in medical data analysis has been to develop models for typical classification problems, where an object is related to a single class from a set of mutually exclusive categories. There is, nevertheless, another task in which classes are not mutually exclusive but are presented in the form of multilabel assignments. Let us say we have label sets *C* =  {*C*_*i*_}, *i* = 1…|*C*|, in multiclass classification (MLC); each example belongs to a single class *C*_*i*_. The labels are mutually exclusive, and data cannot be related to more than one class. Multilabel classification requires specialized machine learning algorithms to predict multiple mutually nonexclusive labels or categories since examples are associated with a set of labels *Y* ⊆ *C* [21]. Problem transformation [22–24] and algorithm adaptation [25–27] are the broadly used techniques to deal with multilabel classification problems.

Though deep learning is growing popular in its performance, serious thought is necessary to develop a specific architecture that is well suited to the nature of the analyzed data to create an efficient model. Adopting deep CNN models developed for image analysis is not straightforward. They have massive parameters that lead to overfitting and extensive computation. Besides, they do not go with the characteristics of the ECG signal. Therefore, we designed and implemented a lightweight, multireceptive field CNN for the PTB-XL dataset [28] classification in this study.

## 2. Related Work

One of the earliest uses of classical machine learning includes ECG beat classification with the Gaussian RBF kernel support vector machine (SVM) after extracting 20 significant features from the MIT-BIH dataset by the Discrete Wavelet Transform (DWT) and Principal Component Analysis (PCA) [29]. Li et al. [30] developed ventricular fibrillation (VF) and rapid ventricular tachycardia (VT) detection by extracting 14 features from three annotated public domain ECG databases (the American Heart Association Database, the Creighton University Ventricular Tachyarrhythmia Database, and the MIT-BIH Malignant Ventricular Arrhythmia Database). Then they used SVM as a classifier.

The authors in [31] used DWT to denoise the ECG signal first and then Pan-Tompkins [32] for QRS detection. They performed ECG beat segmentation after the QRS detection. Feature extraction is performed from the segmented ECG signal using HOS with ICA and DWT with PCA. The extracted features are fed to SVM and NN for classifying the MIT-BIH AD dataset into five types of ECG beats (nonectopic (*N*), supraventricular ectopic (*S*), ventricular ectopic (*V*), fusion (*F*), and unclassifiable and paced (*U*) beats). The average accuracy of 99.57% and 99.56% is achieved with SVM and NN, respectively, on the MIT-BIH AD dataset. Li and Zhou [33] developed an ECG classification on the MIT-BIH Arrhythmia Database. First, they decomposed the ECG signals using wavelet packet decomposition (WPD) and then calculated the entropy as representative features from the decomposed coefficients. Random Forest is used as a classifier and achieves good test time and accuracy. This study indicates that entropy and RR intervals perform better than the ICA-RR and DWT-RR.

Celin and Vasanth [34] used low pass, high pass, and Butterworth filters to preprocess ECG signals. After preprocessing, R-peak detection is performed, and features such as mean, standard deviation, root mean square, pulse transit time, and pulse rate variability are extracted. These features are fed to the Naive Bayes classifier to classify ECG signals as normal and abnormal.

Billeci et al. [35] proposed a multiclass SVM classifier for detecting normal rhythm, atrial fibrillation, and other arrhythmias from ECG recordings on a smartphone device. Since the smartphone device is not suitable for multilead recording, a single lead point of care device, AliveCor^TM^, was used to record the signals for the smartphone. They used 30 features extracted from the RR intervals analysis, analysis based on P wave absence (PWA), and frequency spectrum analysis (FSA) for training their algorithm. They achieved an *F*_1_ score of 0.83 on the PhysioNet Challenge and 0.98 on the MIT-BH ADF database.

In paper [36], the MIT-BIH Arrhythmia Database was used to classify heartbeats into four types using an ensemble-based support vector machine (SVM) classifier. SVM, Random Forest (RF), *K*-Nearest Neighbours (KNN), and Long Short-Term Memory network compared the findings with the ensemble-based SVM classifiers. Wavelets, high order statistics, R-R intervals, and morphological features are the four features retrieved from ECG signals that the classifiers use. The best result was obtained using an ensemble of SVMs with an overall accuracy of 94.4%.

Sraitih et al. [37] performed normalization using min-max normalization and then denoised the ECG signal using the Butterworth digital filter with a cutoff frequency of 0.25 Hz and a filter order of 3. The signal is then sampled at 0.66 s segments for each beat, *t* = 0.33 s after and before the R-peak position. Without any feature extraction, the results from the segmentation process are directly fed to four supervised classifiers: SVM, KNN, RF, and the ensemble of these three classifiers. These four methods were investigated in classifying the ECG beats into Normal (NOR), Left Bundle Branch Block (LBBB), Right Bundle Branch Block (RBBB), Premature Atrial Contraction (PAC), and Premature Ventricular Contraction (PVC) beat from MIT-BIH Database. The study emphasized that, by applying no detailed data preprocessing or feature engineering methods, SVM outperformed the other practices by achieving an accuracy of 83%.

Despite the excellent performance achieved by the classical machine learning approach on a small dataset, being cheaper for development and easier for interpretation, most of the research on automatic detection of abnormalities on ECG focused on detecting only a single abnormality or a few abnormalities with the most popular abnormalities, including arrhythmia, ventricular fibrillation, and tachycardia. Deep learning is more preferred than classical machine learning because it scales effectively with data, does not need feature engineering, and is adaptable and transferable [38]. Applying RNN, CNN, and DNN for computer-aided cardiac abnormality detection has become famous as the ECG dataset grows in volume. The PhysioNet/CinC Challenge datasets [39] are among the popular publicly available ECG datasets.

Izci et al. [40] proposed a deep learning-based approach for detecting five distinct forms of ECG arrhythmias (*N*, nonectopic or paced beats; *S*, supraventricular ectopic beat; *V*, ventricular ectopic beat; *F*, a fusion of ventricular and *Q*-healthy rhythm, pace beat, or fusion of a paced and a normal or beat that cannot be classified). In segmentation processing, ECG signals are converted into ECG beats. Each beat of the 1D ECG signal is then transformed into a 2D grayscale image as input data for the proposed 2D-CNN structure. This model has attained high-performance measurements for diagnosing five different arrhythmic heartbeats with an accuracy of 97.42% on the MIT-BIH Arrhythmia Database. Similarly, Zhao et al. [41] modified the ResNet34 deep learning architecture to have a 1D filter instead of the 2D filter to make it suitable for a 1D ECG signal. They achieved an average accuracy of 98.6% in categorizing heartbeats from the ECG into the five forms of ECG arrhythmia on the MIT-BIH Arrhythmia Database.

Khatibi and Rabinezhadsadatmahaleh [42] used features extracted by pretraining deep learning models (ResNet50 and VGGNet16) and handcrafted features (RR features) from the MIT-BIH database for training different classifiers. They used the KNN algorithm for feature engineering. The pretraining deep learning model extracts features and reduces them by calculating the linear correlation coefficient and removing features with less than some value determined by trial and error. The SVM with polynomial kernel was the best performing classifier with a classification accuracy of 99.7% in classifying heartbeats into Normal (NOR), Premature Ventricular Contraction (PVC), and Premature Atrial Contraction (PAC) beats.

Teplitzky et al. [43] used a deep learning-based BeatLogic platform designed by fusing two deep learning networks, RhythmNet and BeatNet, which are designed based on the ResNet architecture, to annotate ECG graphs. The RhythmNet architecture is responsible for the detection and classification of sinus rhythm (Sinus), atrial fibrillation/flutter (AFib), supraventricular tachycardia (SVT), junctional rhythm, second-degree heart block type 1 (BII1), second-degree heart block type 2 (BII2), third-degree heart block (BIII), and others. In contrast, BeatNet architecture is for detecting ventricular rhythms, IVCD, and Pause. The proposed method achieved a 0.95 *F*_1_ score for atrial fibrillation/flutter, ventricular tachycardia, ventricular bigeminy, ventricular trigeminy, and third-degree heart block detection.

On the PTB-XL dataset, Strodthoff et al. [44] provided benchmarking tasks ranging from ECG statements prediction from various subsets of ECG statements and label granularity to age and sex prediction. They adapted state-of-the-art deep learning models for image classification to the ECG context. The authors also claimed that modern ResNet-based or Inception-based CNN architectures performed best, particularly the newly proposed ResNet variant XResNet1d. Still, recurrent architectures are also competitive for a particular prediction task. Modern ResNet-based or Inception-based CNN architectures, particularly the recently proposed ResNet variant XResNet1d101, perform best with a macro-averaged AUC of 93.5%, 92.9%, and 92.8% for 44, 23, and 5 classes, respectively, but recurrent architectures are also competitive for specific prediction tasks.

Śmigiel et al. [45] developed a lightweight CNNs model and integrated it with entropy, which is calculated after the signal is converted to a spectrogram. They claimed that using the entropy features significantly improved the performance of their model on the PTB-XL database. They also claim that adding QRX complexes features extracted from the signal substantially enhances performance in the study they carried out in paper [46]. The authors in [47] proposed a neural network trained for conducting Few-Shot Learning (FSL) classification and proved that FSL-based classification is more accurate than the softmax-based classification. The authors in [48] tried to address the challenges of cross-institutional algorithm evaluation using transfer learning and frequency domain CNN. They demonstrated their work for atrial fibrillation classification on the PTB-XL dataset and two additional datasets from different institutions. Another study that uses the PTB-XL dataset to build a model for diagnosing normal and abnormal ECG with adaptive feature was conducted by Zhu et al. [49]. The model has three modules: (1) convolutional neural network-based feature extraction module, (2) recursive feature elimination based on the weights of the features, and (3) a fully connected layer for classification.

There are some challenges in developing a machine learning model for cardiac abnormality classification from the ECG datasets. Firstly, no ECG dataset is available with a massive sample number like the ImageNet dataset. This property leads to overfitting if an intense CNN architecture is used for the ECG datasets. Secondly, the nature of information context for ECG and image is very different. Hence, while designing a CNN model for ECG analysis, attention must be given to exploiting the nature of the ECG datasets to improve performance. The other challenge is that ECG datasets are likely to have classes imbalanced. Cardiac abnormalities are likely to have biased distributions because most severe diseases occur rarely but are essential [50].

Even though there is a noticeable improvement in deep learning performance in classifying abnormalities on ECG signals, the focus is mostly on arrhythmias and there is lack of universality. Emphasis must also be given to the class imbalance in the ECG datasets, and the model developed should consider the signal properties of ECG data.  Table 1 summarizes the essential findings and limitations of each related work.

## 3. Materials and Methods

This section covers the techniques and workflow employed to design and implement multireceptive field CNN for ECG signal classification. The research methodology described in this paper is demonstrated in Figure 2. First, dataset preprocessing and preparation will be discussed. After that, the detailed design of the MRF-CNN will be addressed. Finally, the model will be evaluated using macro-averaged metrics, and a comparison with the existing methods will be provided.

### 3.1. Dataset

The proposed method is tested on the PTB-XL ECG dataset [28]. It is the most significant freely accessible clinical 12-lead ECG waveform. The waveform data in the dataset was collected for seven years between 1989 and 1996. Twelve-lead readings with reference electrodes on the right arm are provided. Each record was annotated with a reporting string converted into a standardized set of SCP-ECG statements [51]. The dataset contains 21837 12-lead ECG records with *F*_1_ of 0 seconds from 18885 patients, among which 48% is for female patients, and 52% is for male patients, and it covers an age range from 0 to 95. PTB-XL dataset is complex because it covers a wide age range (0–95), and it is a multilabel dataset, where diagnostic labels are further aggregated into superclasses and subclasses.

In the dataset, there are 71 unique classes, given in Table 2. The 71 classes comprise 44 diagnostic, 19 form, and 12 rhythm classes. The diagnostic category can be further arranged hierarchically into a superclass and subclass. The waveform files are saved in a format with 16-bit precision, at a resolution of 1 *μ*V/LSB and a sampling frequency of 500 Hz and 100 Hz. Since the signal was recorded for 10 seconds, there will be 1000 discrete values for 100 Hz and 5000 for 500 Hz per record.

We have employed two approaches in the data preprocessing stage: windowed and nonwindowed. In the windowing data preprocessing, 2.5 seconds of window size with 50% overlap are used as discussed in [44]. On the other hand, for the nonwindowing approach, the whole record is fed to the model without any segmentation. We have also experimented by removing classes with less than 20 sample numbers. The dataset was divided into training, testing, and validation sets in 70%, 15%, and 15%, respectively. Finally, while standard normalization is performed on the raw signal, the multilabel is converted to multihot using the scikit-learn MultiLabelBinarizer.

### 3.2. Proposed Multireceptive Field CNN

Multireceptive field CNN is a deep learning architecture in which we have multiple receptive fields to extract features from the inputs [52]. Wang et al. [53] proposed a 1D multiscale CNN for bearing fault diagnosis. Their model uses three feature extractors with different convolutional kernel sizes, enabling the mode to learn from the varying size of the receptive field. Cui et al. [54] proposed an end-to-end multiscale CNN model that considers the fact that features in the time-series dataset often appear at different time scales. Applying multireceptive field CNN with dilated and multiple kernels also works well for semantic segmentation of medical images [55].

Every single point in a feature map of a CNN-based model is generated via a receptive field. For example, as illustrated in Figure 3, the receptive field (3 × 3, nine pixels) given as green pixels in layer 1 produces a green pixel in layer 2. On the other hand, the receptive field in 1D-CNN will be 1-dimensional, as depicted in Figure 4. The primary purpose of the convolutional neural network is to detect local low-level features in a given signal. The receptive field of CNN architecture directly relates to the filter size used in the architecture, as explained in Section 1. For example, if we use a kernel size of 3, we necessarily say that low-level features are 3 points wide. We can design a multireceptive field CNN using two ways. The first is by using multiple kernels of different sizes. The second is using a fixed-size kernel with a varying dilation rate to obtain multiple receptive fields [55]. Figure 4 describes the effects of kernel size and dilation rate. In (a), a kernel size of 5 and 7 is used with dilation rate of 1, resulting in 5 and 7 broad receptive fields, respectively. In (b), the same kernel size is used but with a dilation rate of 2, resulting in 9 and 13 receptive fields, respectively. Therefore, to increase the receptive field size, we can increase either the kernel size or dilation rate.

As shown in Table 3, features in ECG signals are found at different sizes (interval or duration). Hence, we have proposed a multireceptive field 1D-CNN model for automatic multilabel classification of the 12-lead ECG dataset. CNN architecture that ensures its receptive field covers the entire relevant input signal region is designed and tested to be robust compared to the existing deep learning models for PTB-XL dataset classification. Therefore, multiple filters with sizes of 7 and 5 with dilation rates of 1 and 2 and a filter size of 1 with a dilation rate of 1 are used in the proposed model. These kernel sizes are chosen because the ECG signal should capture different interval and segment lengths. Having kernels of different sizes enables the model to capture various features that can discriminate one class of ECG from another. The network facilitates the ability to look into multiple fields simultaneously. Most studies regarding the classification of ECG signals are based on a receptive field generated by a fixed kernel length. However, our work shows generating both small and large receptive fields can improve performance and detect local features of varying sizes. It also enhances the feature discriminability and robustness according to the verification of the experiment carried out in this study.

Therefore, detecting appropriate discriminative features requires a kernel of different sizes instead of a fixed one. The proposed model (Figure 5) has large and small blocks to see features from larger and smaller receptive fields. The LargeBlock contains five 1D convolutions (7 × 1 and 5 × 1 kernels with dilation rates of 1 and 2 and an additional filter of 1 × 1 with a dilation rate of 1) followed by batch normalization, activation, and max pooling. The SmallBlock is identical to the LargeBlock, except that the filter sizes are 7 × 1, 5 × 1, and 1 × 1, and there is a dropout with a 0.20 rate after each max pooling. Finally, global average pooling is used in the fully connected layer instead of flattening. The global average pooling is followed by one dense layer and the final output layer. Global average pooling has an advantage over the flattening layer as more native to the convolution structure, and there is no parameter to optimize; thus, overfitting is avoided at this layer [56].

Since the PTB-XL dataset is multilabel, the CNN must be configured to support the MLC task. Therefore, Sigmoid is used as an activation function for the output layer. The likelihood of an instance belonging to a particular class is calculated using Sigmoid. The label is true if the probability is more than a given threshold (0.5 in this study). In the layers other than the output layer, Leaky ReLU is used. The most widely used loss function for MLC is binary cross-entropy [57]. The factor that leads to selecting a cross-entropy loss function is the output layer activation function, Sigmoid. The binary cross-entropy computes the cross-entropy loss between the input label and the predicted output probability of the model.

The model's number of parameters is few as it is lightweight and special consideration is taken to minimize the computational resource requirement of the model. To reduce the numbers of parameters and dimensions of inputs of the network's layers, we used max pooling and 1 × 1 convolution filters. The max pooling operation minimizes the input width by two after each layer. Concatenation of each feature map increases the channel number enormously. Hence, the 1 × 1 Conv reduces the channel number.

### 3.3. Evaluation

In most classification tasks, the accuracy is used as an evaluation matrix. It indicates the ratio of correctly classified labels to the total number of classifications. However, it does not tell the whole story in some cases. Hence, it may lead to a wrong conclusion about the model. Calculating the confusion matrix is advised to get the entire idea about the model's performance.

A confusion matrix is a tabular representation of the results that describe the overall performance of the classification model, depicted in Table 4. The essential operation is a confusion matrix that accepts the label of test data, compares it with the predicted output from the classifier model, and gives the result score for each class [58]. Metrics like AUC, recall, precision, and *F*_1_ score are defined from the confusion matrix. They give us a more accurate measure of what is going on than accuracy.

Accuracy is the number of correct predictions divided by the total number of samples in the dataset. *F*_1_ score is used to create a balance between precision and recall, and it is sometimes referred to as the F score or F measure. Precision can be obtained by dividing the true positive by the number of positive and false negative values. In contrast, recall is obtained by dividing the true positive by submitting true positive and false negative values.

(1) $$\begin{array}{c} \text{FalsePositiveRate}=\frac{FP}{\left(TN+FP\right)}, \end{array}$$

(2) $$\begin{array}{c} \text{TruePositiveRate}=\frac{TP}{\left(TP+TN\right)}. \end{array}$$

The other metric used to evaluate the model presented in this study is AUC, calculated from ROC (receiver operating characteristic curve). ROC is a graph plotting a true positive rate (2) versus a false positive rate (1) at different classification thresholds. The lower the classification threshold is, the more items the classifier classifies as positive. AUC represents the area under the ROC curve.

(3) $$\begin{array}{c} \text{Accuracy}=\frac{TP}{\left(TP+TN+FP+FN\right)}, \end{array}$$

(4) $$\begin{array}{c} \text{Precision}=\frac{TP}{\left(TP+FP\right)}, \end{array}$$

(5) $$\begin{array}{c} \text{Recall}=\frac{TP}{\left(TP+FN\right)}, \end{array}$$

(6) $$\begin{array}{c} F_{1}\text{Score}=2*\frac{\text{Precision}*\text{Recall}}{\left(\text{Precision}+\text{Recall}\right)}. \end{array}$$

In multilabel classification (MLC), a prediction could be completely accurate if the predicted labels *P* are the same as the ground truth labels *Y*, partially accurate if *Y* ∩ *Z* ≠ ∅, or utterly wrong if *Y* ∩ *Z* = ∅. The multilabel classification (MLC) evaluation metrics are divided into example-based and label-based metrics. Performance is calculated for each data instance and averaged over the whole dataset with example-based metrics. On the other hand, label-based metrics measure each label's performance separately before averaging across classes [59]. Hence, in this study, label-based macro-averaged accuracy, AUC, recall, precision, and *F*_1_ score are used to evaluate the performance of the proposed model.

The label-based evaluation considers every label separately, reducing MLC to a binary classifier for a particular label, with four possible prediction outcomes: TP, FP, TN, and FN. Accuracy, precision, recall, and *F*_1_ score are calculated by equations (3)–(6): label-based classification metrics for the classifier H and dataset *D*_*t*_ could be obtained using macro or micro averaging techniques. Let B be any of the measures defined by equations (3)–(6). *B*_macro_ (*H*, *D*_*t*_) and *B*_micro_ (*H*, *D*_*t*_) are calculated as follows [60]:

(7) $$\begin{array}{c} B_{\text{macro}}\left(H,D_{t}\right)=\frac{1}{q}\sum_{j=1}^{q}B\left(TP_{j},FP_{j},TN_{j},FN_{j}\right),\\ B_{\text{micro}}\left(H,D_{t}\right)=B\left(\sum_{j=1}^{q}TP_{j},\sum_{j=1}^{q}FP_{j},\sum_{j=1}^{q}TN_{j},\sum_{j=1}^{q}FN_{j}\right), \end{array}$$

where *j* = 1,…, *q* and *q* represents the number of labels in the classification task.

On the other hand, the example-based evaluation metrics are found by considering each instance's hit and miss ratio regardless of the label and averaging the entire test set. Example-based precision, recall, and *F*_1_ score are defined as follows:

(8) $$\begin{array}{c} {\text{Precision}}_{EB}=\frac{1}{N}\sum_{i=1}^{N}\frac{\left|Y_{i}\cap P_{i}\right|}{\left|P_{i}\right|},\\ {\text{Recall}}_{EB}=\frac{1}{N}\sum_{i=1}^{N}\frac{\left|Y_{i}\cap P_{i}\right|}{\left|Y_{i}\right|},\\ F_{1}{\text{Score}}_{EB}=\frac{2*{\text{Recall}}_{EB}*{\text{Precision}}_{EB}}{{\text{Precision}}_{EB}+{\text{Recall}}_{EB}}, \end{array}$$

where *Y*, *P*, Recall_*EB*_, and *Precision*_*EB*_ are ground truth, prediction results, example-based recall, and example-based precision, respectively, for *i* = 1,2,…, *N* and *N* represents number of examples.

Therefore, in this research, we used macro-averaged precision, recall, *F*_1_ score, AUC, and accuracy to measure how the proposed model performed. Example-based *F*_max_ is also used. Maximum *F*_1_ score (*F*_max_) is an *F*_1_ measure at a threshold that gives a maximum value rather than 0.5. Other than these metrics, training AUC, validation AUC, training loss, and validation loss were used to measure model performance during training.

Applying the default evaluation metrics of unskewed data to skewed data can have a negative effect on the model's performance. Using standard metrics in the imbalanced dataset can lead to suboptimal classification models and might produce misleading conclusions, since these measures are insensitive to the skewed dataset. The main problem of imbalanced datasets is that they are often associated with a user preference bias towards the performance of underrepresented classes in the available data sample [61]. When a dataset is balanced, using accuracy is usually a good start. It will help if accuracy is not used when a heavily imbalanced dataset is considered. Therefore, the *F*_1_ score and AUC are appropriate for a class imbalance. The intuition is that the false positive rate for highly imbalanced datasets is ruined due to many true negatives. If we care about true negatives as much as true positives, AUC and *F*_1_ scores are used [62–64].

## 4. Results and Discussion

ECG signal classification is performed using the proposed model in the experiment, and the model's performance is compared with the existing model. From the experiments carried out in this study, the optimal hyperparameters are obtained using grid search. Although the epoch number used is 100, early stopping with a tolerance of 10 is used to get the best network parameters. RMSProp optimizer, 128 batch size, and 0.0001 learning rate are the optimal values of the parameters. A summary of the hyperparameter setting is found in Table 5.

Based on the previous works of the literature on the PTB-XL dataset classification, we have tested our model under two scenarios. The first scenario is that classes with a sample number of less than 20 are removed from the dataset as is done in [45–47]. The second scenario is working on the whole dataset without removing any classes. However, the sliding window approach is used to train the classifier on random segments of fixed length (2.5 seconds) taken from the entire record as is done in [44]. In this case, during the test time, the signal is divided into segments of 2.5 seconds with 50% overlap and obtains model predictions for each segment. These predictions are then aggregated using the element-wise maximum to produce a single prediction for the record.

We have compared the performance of the proposed model under both scenarios with the existing model. Under the first case, the proposed model has a significant performance improvement compared to the architecture in [45–47] as portrayed in Tables 6–8. The performance gain in evaluation metrics (accuracy, precision, recall, *F*_1_ score, and AUC) is significant, and the proposed model has fewer parameter numbers.

Similarly, the model performance under the second scenario is evaluated and found to be the same as that of [44] with a significant improvement in the parameter number (Table 9). In [44], the model with the least parameter number is FCN-Wang with 311,700 total parameters. This model has a performance of 0.926, 0.928, and 0.930 label-based macro-averaged AUC for the diagnostic, subdiagnostic, and superdiagnostic classes, respectively. It also produces 0.735, 0.762, and 0.823 example-based *F*_max_ for the diagnostic, subdiagnostic, and superdiagnostic classes, respectively. The proposed model exhibits a nearly similar performance in terms of AUC and *F*_max_ scores; however, the number of parameters decreases by five. The proposed model has 0.930, 0.922, and 0.927 AUC and 0.720, 0.743, and 0.816 *F*_max_ with 59,060 number of parameters.

Moreover, Table 10 shows the result without using the sliding window concept, using the whole signal as input to the model. The performance drop indicates that using the sliding window concept can improve performance. In the sliding window approach, a segment of 2.5 seconds is taken from the record and used for prediction. The advantage of this approach is that it generates additional data and can be used as a data augmentation technique, leading to a performance gain. Nevertheless, in some conditions of cardiac abnormalities, the features that indicate a given situation may manifest at a specific location but not all over the signal.

The flaw in the current work that we decided to mitigate is using a fixed-size kernel, which only generates a receptive field with a fixed size. What we did was examination using numerous receptive fields of various sizes rather than just one large or small receptive field. Using this method, the model can investigate several nearby places at once. According to the experimental findings (Tables 7–9), CNN with multireceptive fields has improved performance.

## 5. Conclusion

The electrical activity produced during the heartbeat is measured and recorded by an ECG. Cardiologists can interpret the ECG machine's signals and determine the heart's health condition and related causes of ECG signal abnormalities. However, cardiologist shortage is a challenge in developing countries and developed countries. On the other hand, the experience of a cardiologist matters in the accurate interpretation of the ECG signal, as the interpretation of ECG is quite tricky even for experienced doctors. Therefore, developing computer-aided ECG interpretation is required for its wide-reaching effect.

CNN-based deep learning is more effective than classical machine learning detection algorithms in classification performance. 1D-CNN is being widely used for CVDS detection from ECG signals. However, adopting a deep learning model designed for computer vision can be problematic because of its massive parameters and the need for many samples to train. In many detection tasks ranging from semantic segmentation of medical images to time-series data classification, multireceptive field CNN has improved performance. Notably, the nature of the ECG dataset made performance improvement possible by using a multireceptive field CNN. Using MRF-CNN, it is possible to design a model that considers semantic context information within ECG signals with different sizes. As a result, this study has developed a lightweight multireceptive field CNN architecture for ECG analysis. The proposed MRF-CNN architecture can improve the performance of ECG signal classification. 1 × 1 convolution and max pooling reduce the numbers of parameters and dimensions of inputs to the network layer. The 1 × 1 convolution controls the depth of the input volume as it propagates to the following layers and introduces nonlinearity to the network; max pool downsamples the input for dimension reduction and makes the model feature extraction process be rational/position invariant. We have achieved a 0.72 *F*_1_ score and 0.93 AUC for superclasses, a 0.46 *F*_1_ score and 0.92 AUC for subclasses, and a 0.31 *F*_1_ score and 0.92 AUC for the diagnostic classes of the PTB-XL dataset by removing classes with less than 20 sample number.

## 6. Future Work

ECG dataset suffers from class imbalance as the distribution of cardiac abnormalities is not similar. For future work, we recommend using a generative adversarial network and other one-dimensional data augmentation techniques to generate ECG signals to tackle the data imbalance issue. We also recommend combining wavelet transform and raw signal fusion to get broad feature representation and then improving classification performance.

## Figures and Tables

**Figure 1:** ECG waves, segments, and intervals [4].

**Figure 2:** Framework of the proposed methodology.

**Figure 3:** Receptive field for 2-dimensional convolutional neural network [20].

**Figure 4:** Multireceptive field (a) using two kernels with a dilation rate of 1 and (b) two kernels with a dilation rate of 2, while the dots represent data points in a given signal.

**Figure 5:** The proposed model architecture: the picture in (a) indicates the proposed lightweight and multireceptive field CNN architecture; the LargeBlock and SmallBlock in (b) have different kernel size and dilation rates to build the multireceptive field CNN. The model has six layers: five convolutional layers and one fully connected layer. Finally, Sigmoid is used as an activation function for class probability prediction.

**Table 1:** Literature summary table.

Author(s)	Dataset	Purpose	Method	Key findings	Limitations
Thanapatay et al. [29]	MIT-BIH Arrhythmia Database	ECG beat classification	Discrete wavelet transform (DWT) and Principal Component Analysis (PCA) to extract 20 principal features and SVM for classification	The classifier achieved 99.6% in classifying beats	It is only for beat classification, and it is based on image processing techniques
Billeci et al. [35]	MIT-BIH AF Arrhythmia Database	Classification in short ECG recordings acquired using a smartphone device	51 features extracted and LS-SVM is used for classification	Performance for normal rhythm 0.98, AF rhythm 0.99, and global 0.98 *F*_1_ score	Atrial fibrillation classification only
Khatibi and Rabinezhadsadatmahaleh [42]	MIT-BIH Arrhythmia Database	Arrhythmia detection from beat classification	Features extracted by pretraining ResNet50, VGGNet16, and handcrafted features (RR features). SVM, KNN, Decision Trees, and Random Forests are used for classification	It has a lower computational need for training than a deep learning model built from the ground up, and it outperforms classical machine learning	The model has millions of parameters, and it only detects arrhythmias
Zhao et al. [41]	MIT-BIH Arrhythmia Database	Patient-specific classification of arrhythmias	ResNet34 deep learning architecture with a 1D filter	Average accuracy of 98.6% in the categorization of heartbeats	Model with millions of parameters and it overfits quickly
Śmigiel et al. [45]	PTB-XL database	Subclasses of diagnostic categories in the PTB-XL	CNN with six layers with entropy as an additional feature	0.698 accuracy, 0.332 *F*_1_ score, and 0.815 AUC	Low accuracy, *F*_1_ score, and AUC
Śmigiel et al. [46]	PTB-XL database	Classification of 2, 5, and 20 classes of heart diseases in the PTB-XL dataset	CNN to perform the encoding of a single QRS complex with the addition of entropy-based features	Adding entropy-based features and extracted QRS complexes to the raw signal is beneficial	Low accuracy, *F*_1_ score, and AUC
Pałczyński et al. [47]	PTB-XL database	Training deep CNN to recognize 2, 5, and 20 different heart disease classes from the PTB-XL dataset	Achieved better results in classifying five other disease classes than softmax-based counterparts	Determining the Few-Shot Learning (FSL) applicability for ECG signal proximity-based classification	Low accuracy, *F*_1_ score, and AUC
Zhu et al. [49]	PTB-XL database	Classifying ECG signal into abnormal and normal	CNN as feature extraction module, recursive feature elimination, and fully connected layer for final classification	0.889 accuracy and 0.904 *F*_1_ score	It is only abnormality detection, no further effort to identify specific heart disease from the signal

**Table 2:** Hierarchical arrangement in the diagnostic class of the PTB-XL dataset.

Superclasses	Subclasses	All diagnostic classes	Description
CD	IRBBB	IRBBB	Incomplete Right Bundle Branch Block
	IVCD	IVCD	Nonspecific intraventricular CD
	CRBBB	CRBBB	Complete Right Bundle Branch Block
	CLBBB	CLBBB	Complete Left Bundle Branch Block
	LAFB/LPFB	LAFB	Left anterior fascicular block
		LPFB	Left posterior fascicular block
	WPW	WPW	Wolff-Parkinson white syndrome
	ILBBB	ILBBB	Incomplete Left Bundle Branch Block
	_AVB	3AVB	Third-degree AV block
		2AVB	Second-degree AV block
		AVB	First-degree AV block

HYP	LVH	LVH	Left ventricular hypertrophy
	LAO/LAE	LAO/LAE	Left atrial overload/enlargement
	RVH	RVH	Right ventricular hypertrophy
	RAO/LAE	RAO/LAE	Right atrial overload/enlargement
	SEHYP	SEHYP	Septal hypertrophy

MI	AMI	INJLA	Subendocardial injury infarction
		ASMI	Anteroseptal myocardial infarction
		INJAL	Subendocardial injury in the anterolateral leads
		AMI	Anterior myocardial infarction
		ALMI	Anterolateral myocardial infarction
		INJAS	Subendocardial injury in anteroseptal leads
	LMI	LMI	Lateral myocardial infarction
	IMI	IPLMI	Inferoposterolateral myocardial infarction
		IPMI	Inferoposterior myocardial infarction
		ILMI	Inferolateral myocardial infarction
		INJIL	Subendocardial injury in inferolateral leads
		IMI	Inferior myocardial infarction
		INJIN	Subendocardial injury in lateral leads
	PMI	PMI	Posterior myocardial infarction

NORM	NORM	NORM	Normal ECG

STTC	STTC	NDT	Nondiagnostic T abnormalities
		DIG	Digitalis effect
		ANEUR	ST-T changes compatible with ventricular aneurysm
		EL	Electrolytic disturbance or drug
		LNGQT	Long QT-interval
	NST_	NST_	Nonspecific ST changes
	ISC_	ISC_	Nonspecific ischemic
	ISCI	ISCIN	Ischemic in inferior leads
		ISCIL	Ischemic in inferolateral leads
	ISCA	ISCAL	Ischemic in inferior leads
		ISCAS	Ischemic in anteroseptal leads
		ISCLA	Ischemic in lateral leads
		ISCAN	Ischemic in anterior leads

**Table 3:** Typical amplitudes and durations of ECG signal for adult.

Wave	Amplitudes (mV)	Durations (seconds)
P wave	0.10–0.30	0.04–0.12
PR interval	120–200	0.12–0.20
QRS interval	1-2	0.05–0.10
R wave	0.2–1.7	<0.07
ST interval	—	0.12–0.32 (mean)
ST segment	—	0.24 (mean)
T wave	0.05–0.80	0.10–0.25
QT interval	—	0.30–0.40
PQRST	—	0.42–0.60

**Table 4:** Confusion matrix table for binary class classification.

		Prediction result	
		Positive	Negative
Actual result	Positive	True positive (TP)	False positive (FP)
	Negative	False negative (FN)	True negative (TN)

**Table 5:** Hyperparameter values.

Hyperparameters	Value
Number of epochs	100
Dropout rate	0.20
Loss function	Binary cross-entropy
Batch size	16, 32, 64, 128, and 256
Optimizer	Adam, SGD, and RMSProp
Activation function	Leaky ReLu (*α* = 0.01) and Sigmoid for the final layer
Learning rate	0.01, 0.001, 0.0001, and 0.00001

**Table 6:** Results of the proposed model on the dataset after removing classes with sample number of less than 20 and feeding the whole signal to the model without using any sliding window approach.

Class number	Accuracy	Precision	Recall	*F*_1_ score	AUC
5 (superdiagnostic)	0.897	0.73	0.71	0.72	0.93
20 (subdiagnostic)	0.962	0.42	0.56	0.46	0.92
41 (diagnostic)	0.98	0.28	0.31	0.29	0.92

**Table 7:** Comparison of results of the proposed model and those of the existing model for 20 class number.

Model	Acc	Prec	Recall	*F*_1_ score	AUC	Total param
[45]	0.765	0.355	0.339	0.332	0.815	58,664
[46]	0.685	—	—	0.336	0.861	—
[47]	0.671	—	—	0.324	0.844	—
Proposed	0.962	0.420	0.560	0.460	0.920	56,732

**Table 8:** Comparison of results of the proposed model and those of the existing model for 5 class number.

Model	Acc	Prec	Recall	*F*_1_ score	AUC	Total param
[45]	0.765	0.714	0.662	0.680	0.910	58,259
[46]	0.763	—	—	0.683	0.907	—
[47]	0.790	—	—	0.717	0.936	—
Proposed	0.897	0.730	0.710	0.720	0.930	55,277

**Table 9:** Comparison of results of the proposed model and those of the existing model for the diagnostic, subdiagnostic, and superdiagnostic classes number.

Authors/method		Diagnostic		Subdiagnostic		Superdiagnostic		Total parameters
Authors	Method	AUC	*F *_max_	AUC	*F *_max_	AUC	*F *_max_	
[44]	LSTM-BiDir	0.932	0.737	0.923	0.757	0.921	0.815	2,332,564
	XResNet101	0.937	0.736	0.929	0.760	0.928	0.815	1,874,196
	LSTM	0.927	0.731	0.928	0.759	0.927	0.820	905,620
	Inception	0.931	0.737	0.930	0.752	0.921	0.810	509,588
	ResNet-Wang	0.936	0.741	0.928	0.762	0.930	0.823	745,284
	FCN-Wang	0.926	0.735	0.928	0.762	0.930	0.823	311,700
Proposed		0.930	0.720	0.922	0.743	0.927	0.816	59,060

**Table 10:** Result of the proposed model without using the sliding window approach and by keeping the whole classes in the dataset.

Diagnostic		Subdiagnostic		Superdiagnostic		Total parameters
AUC	*F*_max_	AUC	*F*_max_	AUC	*F*_max_	59,060
0.879	0.677	0.904	0.685	0.910	0.783	

## Data Availability

The data linked should be changed to “https://physionet.org/content/ptb-xl/”.
